# Rhamnolipid Biosurfactant against *Fusarium verticillioides* to Control Stalk and Ear Rot Disease of Maize

**DOI:** 10.3389/fmicb.2016.01505

**Published:** 2016-09-21

**Authors:** Siddhartha N. Borah, Debahuti Goswami, Hridip K. Sarma, Swaranjit S. Cameotra, Suresh Deka

**Affiliations:** ^1^Environmental Biotechnology Laboratory, Life Sciences Division, Institute of Advanced Study in Science and TechnologyGuwahati, India; ^2^Department of Biotechnology, Gauhati UniversityGuwahati, India; ^3^Institute of Microbial TechnologyChandigarh, India

**Keywords:** rhamnolipid, *Fusarium verticillioides* FS7, *Pseudomonas aeruginosa* SS14, Zea mays L., biocontrol, scanning electron microscopy, *In planta* activity

## Abstract

Antifungal activity of rhamnolipids (RLs) has been widely studied against many plant pathogenic fungi, but not against *Fusarium verticillioides*, a major pathogen of maize (*Zea mays* L.). *F. verticillioides* causes stalk and ear rot of maize or asymptomatically colonizes the plant and ears resulting in moderate to heavy crop loss throughout the world. *F. verticillioides* produces fumonisin mycotoxins, reported carcinogens, which makes the contaminated ears unsuitable for consumption. In this study, the RL produced using glucose as sole carbon source was characterized by FTIR and LCMS analyses and its antifungal activity against *F. verticillioides* was evaluated *in vitro* on maize stalks and seeds. Further, the effect of RL on the mycelia of *F. verticillioides* was investigated by scanning electron microscopy which revealed visible damage to the mycelial structure as compared to control samples. *In planta*, treatment of maize seeds with a RL concentration of 50 mg l^-1^ resulted in improved biomass and fruiting compared to those of healthy control plants and complete suppression of characteristic disease symptoms and colonization of maize by *F. verticillioides*. The study highlights the potential of RLs to be used for an effective biocontrol strategy against colonization of maize plant by *F. verticillioides*.

## Introduction

*Fusarium verticillioides* (Sacc.) Nirenberg (teleomorph *Gibberella moniliformis* Wineland) is genetically the most intensively studied species in *Fusarium* section *Liseola* (Jurgenson et al., 2002). This fungus is primarily a pathogen of maize (*Zea mays* L.) that causes stalk and ear rot, but has also been reported to cause disease in other crops like sorghum (Palmero et al., 2012). *F. verticillioides* is known to produce fumonisins, a polyketide group of mycotoxins (Marasas, 2001). These mycotoxins have been well studied both in terms of their synthesis and in regard to their effects on animals that consume contaminated grains (ApSimon, 2001). Fumonisins have been implicated in oesophageal cancer in humans and subsequently several carcinogenicity mechanisms have been proposed (Rheeder et al., 1992; Howard et al., 2001). They have also been associated with disruption of sphingolipid metabolism and folate transport and described as a potential risk factor for human neural tube defects (Marasas et al., 2004). Hence the prevention of colonization of *F. verticillioides* in maize has occupied a thrust area in food safety research.

The control measures against *F. verticillioides* are mostly reliant on the use of resistant maize cultivars or cultural practices, but these measures have not been very effective (Munkvold and Desjardins, 1997). Genetically engineered maize carrying the gene for Bt-toxin has been reported to reduce the probability of *F. verticillioides* infections and toxin production under field conditions (Munkvold et al., 1997, 1998). Potential biocontrol measures for preventing the growth of this organism have been reported involving the use of endophytic bacteria (Hinton and Bacon, 1995). However, the endophytic bacterium *Bacillus mojavensis* RRC101, a biocontrol agent for fungal diseases in maize, has been reported to be sensitive to fusaric acid produced by *F. verticillioides* (Bacon et al., 2004). This might result in a reduced efficiency of this bacterium under field conditions thereby necessitating further research to explore other biocontrol alternatives against *F. verticillioides*. In this regard, microbial biosurfactants appear to be an interesting alternative to the use of endophytes as antifungal agents against *F. verticillioides*, as they have not been reported to be affected by fusaric acid in the available literature. Biosurfactants are structurally diverse group of surface active metabolites of microbial origin classified broadly into glycolipids, lipopeptides, neutral lipids, polymeric biosurfactants, fatty acids, and phospholipids (Cameotra et al., 2010). Biosurfactants represent ecological alternatives with distinct advantages over their synthetic counterparts, such as biodegradability, possible production from renewable resources, lower or non-toxicity, high specificity and stability over a wide range of temperature (-18 to 121°C), pH (2–12) and salinity (NaCl concentrations up to 20%; Nitschke and Costa, 2007). One of the most widely studied biosurfactant over the years has been the rhamnolipids (RLs; Abdel-Mawgoud et al., 2010; Randhawa and Rahman, 2014). RLs have been demonstrated to have wide range of applications in bioremediation and enhanced oil recovery (Rahman et al., 2003), pharmaceuticals (Magalhaes and Nitschke, 2013), cosmetics (Piljac and Piljac, 2007); and agriculture owing to their antibacterial and antifungal properties (Abalos et al., 2001; De Jonghe et al., 2005; Perneel et al., 2008; Varnier et al., 2009). However, the use of RLs as antifungal agents against *F. verticillioides* in maize plant under field conditions has not been reported in existing literature.

In the present study, we evaluated the efficacy of RLs as prospective antifungal agents *in vitro* against *F. verticillioides* using maize stalks and seeds. Further, the antifungal effect was also evaluated *in planta* under natural field conditions.

## Materials and Methods

### Microorganisms

The bacterial strain *Pseudomonas aeruginosa* SS14, reported earlier to produce rhamnolipid (RL) biosurfactant, was used in the present study (Borah et al., 2015). This strain was isolated from crude oil contaminated soil of Lakowa in Sivasagar district of Assam, India (27°0′44″ N, 94°51′17″ E; altitude 95 m) and maintained on nutrient agar (NA) slants at 4°C, subcultured every 2 weeks.

The fungal strain *F. verticillioides* FS7 (GenBank accession no. KF031434) was isolated from symptomatically infected stalks obtained from a maize field of Tinsukia, Assam, India (27.5° N, 95.37° E; altitude 116 m). The detailed method of isolation has recently been published (Borah et al., 2016). For identification of the strain FS7, the ITS1-5.8S-ITS2 regions of the rDNA were amplified and sequenced. Then, the closely related sequences of *F. verticillioides* strain FS7 were identified using Blast2Go Pro software (Conesa et al., 2005; Gotz et al., 2008) and selecting non-redundant database with a blast e value 1.0E-03 filter. A phylogenetic tree (**Figure 1**) was constructed with the query sequence and with representative sequences of reference strains from NCBI database. The tree was generated using the Neighbor-Joining method (Saitou and Nei, 1987) with a bootstrap value of 2000. The analysis involved 21 nucleotide sequences with a total of 1344 positions in the final dataset. Evolutionary analyses were conducted in MEGA6 (Tamura et al., 2013). The fungus was stored as microconidial suspensions at -80°C in 30% glycerol. The working cultures were maintained in Potato dextrose broth (PDB) and PDA plates at 4°C and were subcultured every 2 weeks.

**FIGURE 1:** **Phylogenetic tree of *Fusarium verticillioides* strain FS7 and its related sequences retrieved from NCBI database**.

### Production, Purification, and Characterization of Biosurfactant

Biosurfactant was produced by *P. aeruginosa* SS14 in mineral salt medium (MSM) containing glucose as sole carbon source (2% w/v). The composition of MSM and cultivation conditions have been previously described in detail (Borah et al., 2015). Biosurfactant produced was extracted using the ethyl acetate method and purified by silica gel column chromatography (Borah et al., 2015).

Fourier transform infrared spectroscopy (FTIR) in attenuated total reflectance (ATR) mode was performed at a resolution and wave number accuracy of 4 and 0.01 cm^-1^, respectively, and 32 scans with correlation for atmospheric CO_2._ The FT-IR spectra were recorded in a Nicolet 6700 FT-IR System (Thermo Scientific, Waltham, MA, USA). Liquid chromatography mass spectrometry (LC-MS) was performed in a 1260 Infinity LC coupled with a 6410 Triple Quad MS (Agilent Technologies, Santa Clara, CA, USA) as described earlier (Borah et al., 2015).

### Antifungal Activity of the Rhamnolipid Sample against *Fusarium verticillioides*

#### *In vitro* Test for Antispore Activity in Potato Dextrose Broth Amended with Rhamnolipid

This test was performed in 96-well microtiter plates using PDB solutions amended with different concentrations of rhamnolipid produced by *P. aeruginosa* SS14 (RL-SS14) as medium for growth of *F. verticillioides* as previously described (Borah et al., 2015). Rhamnolipid (RL) concentrations used were 5, 10, 25, 50, and 100 mg l^-1^ in PDB. A 100 μl of each RL concentration was inoculated with 20 μl spore inoculum (10^7^ cfu ml^-1^) of *F. verticillioides* and incubated at 25°C for 48 h. Commercial rhamnolipid R-95 (Sigma–Aldrich, St. Louis, MO, USA) was used as standard. Percentage inhibition was evaluated by measuring fungal growth (OD_600_) in a Varioskan Flash Multimode Reader (Thermo Scientific, Waltham, MA, USA).

#### *In vitro* Test for Antimycelial Activity in Potato Dextrose Agar Amended with Rhamnolipid

Rhamnolipid (RL) solutions were prepared (w/v in Milli-Q water) at concentrations of 10, 25, 50, 100, 200 mg l^-1^. Then 3.9 g PDA was added to 100 ml of each RL solution and sterilized. Sterilized media were poured into 90 mm Petri plates. Control plates were prepared with PDA in Milli-Q water. A 6 mm plug of *F. verticillioides* FS7 from 10 days old culture was transferred on to the middle of the plates. The plates were then incubated at 25°C. Antagonistic activity was expressed in terms of percentage inhibition of mycelial growth, measured after 10 days of incubation when the control plates were completely covered by mycelia and were compared to the test plates under observation.

#### Scanning Electron Microscopy of Mycelia Treated with Rhamnolipid

This experiment was performed as per the methodology of Yan et al. (2015) with slight modifications. PDB solutions were prepared with and without RLs (200 mg l^-1^). A spore inoculum (100 μl; 10^7^ cfu ml^-1^) was added to the flasks and incubated at 25°C for 7 days on a rotary shaker (200 × *g*). Subsequently mycelia were excised for sample preparation. The mycelia were washed thrice in phosphate buffer (pH 7.0) and then fixed with 2.5% glutaraldehyde in 0.1 M phosphate buffer (pH 7.0) overnight at 4°C, then rinsed three times in phosphate buffer. Each specimen was subjected to dehydration by ethanol solutions with the concentrations of 30, 50, 70, 80, 90, 95, and 100% sequentially for 15 min, respectively. The samples were then mounted on stubs over carbon tape and observed in an FE-SEM (Zeiss, Σ-Sigma, Germany) Scanning Electron Microscope.

#### Test for Antifungal Activity Using Maize Seeds

Maize seeds were surface sterilized as described earlier (Yates et al., 2003). Seeds were placed in sterile plastic cups, covered with 5.25% sodium hypochlorite, agitated vigorously for 10 min, rinsed twice with sterile distilled water, imbibed in fresh sterile distilled water for 4 h at 25°C, heat-treated for 5 min at 60°C, and then rinsed with cool sterile distilled water. Surface sterilized seeds were soaked for 12 h in RL solutions with concentrations 10, 25, 50, 100, and 200 mg l^-1^. Seeds soaked in sterilized water served as controls. Water agar (3% w/v) plates were prepared in triplicates and two seeds per plate were placed inside. Then 100 μl spore suspension of *F. verticillioides* (10^7^ cfu ml^-1^) was added to the seeds and incubated at 25°C for 10 days. Spore suspension was prepared by adding sterile deionized water to PDA plates and the conidia were aseptically dislodged with a sterile inoculating loop into the water. Spore suspensions were then aseptically filtered through a 100 μm nylon mesh to remove mycelial debris. Inhibition of infection of the seeds by *F. verticillioides* was studied and evaluated on an 18 point scale using a modification of the method described by Sharma (2011). The criteria for assignment of scores were as follows: (a) no germination and coat infection – zero point, (b) germinated seed showing coat and radical tip infection – one point, (c) either infected – two points, (d) healthy seed showing germination – three points. A total of 18 points were allotted to six seeds per treatment for maximum inhibition.

#### Test for Antagonism against *F. verticillioides* on Maize Stalks

Maize stalks (cut to a size of 1.5 cm × 0.5 cm) were surface-sterilized for 15 min in a 2% solution of sodium hypochlorite and then rinsed three times with sterile water. Surface sterilized maize stalks were put inside sterile Petri plates containing moistened filter paper. A 100 μl of RL at concentrations of 10, 25, 50, 100, and 200 mg l^-1^ (w/v in dH_2_O) was added onto the stalks in the Petri plates. Sterile dH_2_O was added in case of control plates. The plates were then kept overnight at room temperature. After that 100 μl spore suspension of *F. verticillioides* (10^7^ cfu ml^-1^) was inoculated to above maize stalks and incubated at 25°C. Observation of infection of the maize stalks after inoculation of the fungus was done after 10 days of incubation.

### Plant Bioassays

The commercially available cv. of maize PAC 740 (Advanta Ltd., Hyderabad, India) was selected for the present study. The *in planta* antifungal activity of RL against *F. verticillioides* was evaluated by pot assays set up in earthen pots of size 25 cm × 28 cm (diameter × height). Each pot was filled with 4 kg sterilized soil, artificially infested with the test pathogen by inoculating with 500 ml spore suspension of 10^7^ cfu ml^-1^ prepared in PDB. Control pots were inoculated with sterilized distilled water. *In planta* antifungal effect of RL was evaluated by seed treatment with RL before introduction of the seeds into infected soil. The experiments were conducted in the months of August–November when temperature and humidity ranged between 24–30°C and 75–80%, respectively. Plants were irrigated by flooding with sterilized water at an interval of 2–3 days depending on the observed soil moisture. Each treatment set consisted of four replicate pots with one plant in each pot and the experiment was repeated once.

#### Seed Treatment with Rhamnolipid

Surface sterilized maize seeds were soaked overnight in RL solutions of five different concentrations of 10, 25, 50, 100, and 200 mg l^-1^. Control seeds were soaked in sterilized water. The seeds were subsequently sown in *F. verticillioides* infected soil and kept under natural conditions of light, temperature and humidity. Assessment was made on the basis of seed germination, fruiting and dry biomass compared to those of the control treatments sown in pathogen laden and pathogen free soils. For measuring the dry biomass, plants were carefully removed from the pot keeping the roots intact. The plants were then cleaned with tap water to remove excess soil and then rinsed thoroughly with sterilized water, after which they were dried in the shade for 21 days. The weight of the dried plants were measured and tabulated.

#### Detection of Symptomless Infection of *F. verticillioides* in Experimental Plants

To detect the presence of symptomless infection, asymptomatic stalks were surface sterilized for 5 min in a 2% solution of sodium hypochlorite and washed three times with sterile water. Sterilized stalks were split longitudinally and cut into small arbitrary sizes. These cut stalks were placed inside 90 mm Petri dishes containing sterile PDA medium for isolation of *F. verticillioides*. Culture plates were incubated at 25°C for 5–7 days and observed for the presence of *F. verticillioides* colonies, identified microscopically by conidial morphology.

### Statistical Analysis

The data represent the arithmetic averages and the error bars indicate the standard deviations. Results for the antifungal activity of rhamnolipid (RL) using different concentrations, the effect of RL concentrations on disease inhibition and biomass of plants were analyzed using one-way ANOVA with *Post Hoc* pair wise Least Significant Difference (LSD) comparison at a significance level of 0.05. Statistical analyses were performed using the Statistical Package for the Social Sciences (IBM SPSS Statistics 21.0, IBM Corp, Armonk, NY, USA).

## Results

### Characterization of Biosurfactant

The FTIR spectrum (**Figure 2A**) of the biosurfactant sample, produced by *P. aeruginosa* SS14 grown in the medium containing glucose as carbon source was found to be similar to that of the standard RL R-95 thereby confirming the biosurfactant to be rhamnolipid. The band positions were also found to be in agreement with those previously reported for rhamnolipid (RL) produced by *P. aeruginosa* strains (Pornsunthorntawee et al., 2008). The spectral band at 3391 cm^-1^ corresponds to –OH stretching of the hydroxyl group. The strong absorption peak at 2925 cm^-1^ indicates the presence of –CH aliphatic stretching bands. The presence of ester compounds was confirmed by the characteristic peak observed at 1716 cm^-1^, conforming to –C=O stretching vibrations of carbonyl groups. Observation of –C–O– stretching band at 1038 cm^-1^ confirms the presence of the bonds formed between carbon atoms and hydroxyl groups in the chemical structures of the rhamnose rings.

**FIGURE 2:** **Characterization of biosurfactant (RL-SS14) produced by *Pseudomonas aeruginosa* SS14 using glucose as sole carbon source. (A)** FTIR spectra of RL-SS14 in comparison with standard rhamnolipid R-95, the peaks at 3391, 2925, 1716, and 1038 cm^-1^ correspond to –OH stretching of hydroxyl group, -CH aliphatic stretching, -C = O vibrations of carbonyl groups and –C-O- vibrations, respectively. **(B)** Total ion chromatogram (TIC) of RL-SS14 after LC-MS in positive electrospray ionization mode (+ESI). **(C)** Mass spectrum of the fraction eluting at 4.583 min showing the sodiated adduct of rhamnolipid Rha-C_8_ at m/z 351. **(D)** Mass spectrum of the fraction eluting at 11.454 min, the ions at m/z 351 and 505 correspond to Rha-C_8_ and Rha-C_10_-C_10_, respectively.

The total ion chromatogram (TIC) of the purified biosurfactant (**Figure 2B**) acquired by +ESI-LC confirmed the presence of two compounds in the sample. The corresponding mass spectra (**Figures 2C,D**) revealed the presence of two major compounds at m/z 351 and 505. The m/z values obtained were consistent with the sodiated adduct ion [M – H + 2Na] ^+^ and the [M + H]^+^ pseudo molecular ion of the mono-RLs Rha-C_8_ and Rha-C_10_-C_10_, respectively (Deziel et al., 1999).

#### *In vitro* Antifungal Activity of the Rhamnolipid against *F. verticillioides* FS7

##### Antispore activity in potato dextrose broth amended with rhamnolipid

The rhamnolipid produced by *P. aeruginosa* SS14 (RL-SS14) exhibited an inhibition of >50% (i.e., >IC_50_) using concentrations ≥ 50 mg l^-1^ with 88.32% inhibition at 50 mg l^-1^. A significant increase in the antifungal activity of RL-SS14 was observed with increasing concentration (*F*_4,10_ = 3021.808, *P* = 0.000). Moreover, the activity of RL-SS14 was higher than the standard RL R-95 for each of the concentrations used (*F*_9,20_ = 3087.696, *P* = 0.000; **Figure 3**).

**FIGURE 3:** **Antispore activity in terms of percentage inhibition against *F. verticillioides* FS7 on PDB amended with varying concentrations of rhamnolipid produced by *P. aeruginosa* SS14 (RL-SS14) and standard rhamnolipid R-95 after 48 h of incubation at 25°C.** Error bars represent standard deviations (SD). Different letters indicate significantly different values according to LSD at α = 0.05 (*F*_9,20_ = 3087.696, *P* = 0.000).

##### Antimycelial activity on potato dextrose agar amended with rhamnolipid

The antimycelial activity of rhamnolipid produced by *P. aeruginosa* SS14 (RL-SS14) was evaluated by determining the percentage inhibition of *F. verticillioides* growth on PDA amended with RL-SS14 in different concentrations in comparison to the control after 10 days of incubation at 25°C (**Figure 4**). An inhibition of >50% (i.e., >IC_50_) was obtained by using concentrations ≥ 50 mg l^-1^ with 82.23% inhibition at 200 mg l^-1^. Among all the concentrations, a significant difference was evident in the individual effect of each concentration (*F*_4,10_ = 285.931, *P* = 0.000) indicating a concentration dependent activity.

**FIGURE 4:** **Antimycelial activity in terms of percentage inhibition against *F. verticillioides* FS7 on PDA amended with varying concentrations of rhamnolipid produced by *P. aeruginosa* SS14 (RL-SS14) after 10 days of incubation at 25°C.** Error bars represent SD. Different letters indicate significantly different values according to LSD at α = 0.05 (*F*_4,10_ = 285.931, *P* = 0.000).

##### Scanning electron microscopy

Scanning electron microscopy of the untreated mycelia of *F. verticillioides* revealed normal morphology with even thickness and shape (**Figure 5a**), while the RL-SS14 treated mycelia exhibited irregular shape with uneven surface and breakage. The treated mycelia were severely reduced in thickness as compared to the untreated ones (**Figure 5b**).

**FIGURE 5:** **Scanning electron microscopy micrographs of (a) the untreated mycelia of *F. verticillioides* FS7 and (b) mycelia treated with 200 mg l^-1^ rhamnolipid (magnification at 5000×)**.

##### Test for antifungal activity using maize seeds

The results of the experiment evaluated on the basis of scores allotted per seed for each treatment are presented in **Table 1**. The untreated seeds inoculated with fungal spores [control (-)] failed to germinate in five out of six seeds due to infection and seed rot. However, the seeds treated with RL-SS14 concentrations ≥ 50 mg l^-1^ exhibited healthy symptoms comparable to that of untreated un-inoculated [control (+)] seeds.

**Table 1:** Antifungal activity of rhamnolipid produced by *Pseudomonas aeruginosa* SS14 (RL-SS14) evaluated *in vitro* on maize seeds of cv. PAC740 in comparison to untreated healthy and diseased seeds.

Sample	Number of seeds per score category (n)				
	No germination and seed coat infection (Score = n × 0)	Seed coat and radical tip infection (Score = n × 1)	Either seed coat or radical tip infection (Score = n × 2)	Healthy seed germination (Score = n × 3)	Total score
Control (+)	None	None	None	6	18
Control (-)	5	1	None	None	1
10 mg l^-1^	2	3	1	None	5
25 mg l^-1^	1	2	2	1	9
50 mg l^-1^	None	None	2	4	16
100 mg l^-1^	None	None	1	5	17
200 mg l^-1^	None	None	None	6	18

##### Test for antagonism against *F. verticillioides* on maize stalks

Compared with the untreated and infected control (-ve control), no visible lesions were observed on the stalks treated with 50, 100, and 200 mg l^-1^ of RL-SS14. However, visible fungal lesions were observed on maize stalks treated with 10 and 25 mg l^-1^ (**Figure 6A**).

**FIGURE 6:** **(A)** Photograph showing lesions on maize stalks treated with different concentrations (in mg l^-1^) of rhamnolipid produced by *P. aeruginosa* SS14 (RL-SS14) in comparison to controls, after 10 days of inoculation with spore suspension of *F. verticillioides*. **(B)** Photograph showing (I) fungal mycelia on untreated negative control stalks after 7 days of incubation at 25°C; (II) symptomless stalks of plants from seeds treated with 25 mg l^-1^ RL-SS14 before incubation and (III) mycelial development from the same stalks after incubation; (IV) micrograph showing conidia of *F. verticillioides* isolated from stalks in plate III at 100× magnification; (V) symptomless stalks of plants from seeds treated with 50 mg l^-1^ RL-SS14 after 7 days of incubation at 25°C showing complete absence of fungal growth.

### Antifungal Activity of Rhamnolipid in Plant Bioassays

The results of the *in planta* experiment (**Table 2**) revealed that untreated seeds sown in pathogen free soil (positive control) germinated 4–5 days post sowing (dps) while only one seed out of a total of four germinated (at 9 dps) in case of the seeds sown in the pathogen laden soil (negative control). All the seeds treated with RL-SS14 at a concentration ≥ 50 mg l^-1^ successfully germinated. Initiation of fruiting was observed at around 97 dps for the control plants. Seeds treated with RL-SS14 concentrations of 200 mg l^-1^ exhibited comparable (*F*_1,6_ = 0.080, *P* = 0.787) observations to those of positive control plants, whereas those treated with 50 and 100 mg l^-1^ exhibited significantly earlier fruiting period (*F*_2,9_ = 28.532, *P* = 0.000) of around 87 dps. Delayed germination at 7 dps was observed in two replicates for the seeds treated with 25 mg l^-1^, while only one seed germinated (8 dps) in case of those treated with 10 mg l^-1^. These plants survived but exhibited stunted growth with low biomass and no fruiting.

**Table 2:** Time and percentage of germination of seeds, time of fruiting and biomass of plants after seed treatment with rhamnolipid (RL-SS14) in comparison with negative (untreated seeds in pathogen laden soil) and positive (untreated seeds in pathogen free soil) control.

Sample	Germination of seeds^∗^		Time of fruiting (dps)^∗^	Dry weight (in g)^∗^
	Time (dps)	Percentage (%)		
Control (+) (dH_2_O)	4.25 ± 0.5 a	100 ± 0.0 a	97.75 ± 2.5 b	87.5 ± 10.66 b
Control (-)	9.0 ± 0.0 d	25 ± 0.0 c	NF	29.3 ± 0.0 d
10 mg l^-1^	8.0 ± 0.0 c	25 ± 0.0 c	NF	31.1 ± 0.0 d
25 mg l^-1^	7.0 ± 1.41 b	50 ± 0.0 b	NF	57.5 ± 7.78 c
50 mg l^-1^	4.5 ± 1.0 a	100 ± 0.0 a	87.0 ± 1.83 a	100.25 ± 13.15 a
100 mg l^-1^	4.5 ± 0.58 a	100 ± 0.0 a	87.25 ± 2.5 a	103.75 ± 6.75 a
200 mg l^-1^	4.25 ± 0.5 a	100 ± 0.0 a	97.25 ± 2.5 b	81.25 ± 7.89 b

*^∗^Data are means of four replicates ± SD; NF, no fruiting; dps, days post sowing; different letters within each column indicate significant difference between values according to LSD at α = 0.05; ANOVA was performed for time of germination (F_6,21_ = 45.900, P = 0.000), percentage of germination (F_6,21_ = 4.500, P = 0.004), time of fruiting (F_3,12_ = 26.034, P = 0.000), and dry weight (F_6,21_ = 65.795, P = 0.000).*

#### Detection of Symptomless Infection of *F. verticillioides* in Experimental Plants

The culture plate experiment conducted with symptomless stalks confirmed the presence of *F. verticillioides* in stalks of plants from seeds treated with ≤25 mg l^-1^ of RL-SS14. There was no fungal growth from the cultured stalks of plants from seeds treated with ≥50 mg l^-1^ RL-SS14 (**Figure 6B**).

## Discussion

The biosurfactant used in this study was produced by *P. aeruginosa* SS14 using glucose as the sole carbon source and was characterized to be mono-rhamnolipid with two constituent congeners by FTIR and LC-MS analyses. Previously reported strains of *P. aeruginosa* have been documented to produce a mixture of mono and di-rhamnolipids using glucose as a carbon source (Wei et al., 2005; Wu et al., 2008; Lahkar et al., 2015). Therefore, the production of mono-RL by *P. aeruginosa* SS14 might be strain specific as corroborated by earlier reports (Haba et al., 2003) highlighting that the strain of *P. aeruginosa* plays the most important role in determining the composition of a particular RL sample.

The experiments conducted during the present study revealed a stronger antifungal activity of RL-SS14 than that of R-95 against *F. verticillioides*. This might be attributed to the different congener composition of both the RLs as suggested by Das et al. (2014). The activity of RL-SS14 was observed to be stronger against spores than against mycelia. A higher RL concentration was required to obtain a comparable antimycelial and antispore activity. This result follows a similar trend as reported by Kim et al. (2000) and Deepika et al. (2015) for antifungal effect of RL against *Colletotrichum orbiculare* and *F. oxysporum*, respectively, wherein a higher concentration was required to suppress mycelial growth in comparison to that of the spores. This differential activity might be due to the compositional differences between the cell walls of mycelia and spores (Feofilova et al., 2015). Our work is in agreement with previous reports describing the antifungal activities of RL against other species of *Fusarium* (Kim et al., 2000; Sha et al., 2012; Deepika et al., 2015).

Mycelium is the vegetative structure of a fungus that plays a pivotal role in asexual reproduction and disease progression. Therefore, any damage to mycelial integrity might adversely affect the pathogenicity of a fungus. In this regard, SEM was performed to evaluate the effect of RL on mycelia of *F. verticillioides*. The observations highlighted that the RL-SS14 could significantly alter the morphology of the fungal mycelia. The effect of RLs on mycelial structure of fungi has been reported previously (Perneel et al., 2008; Yan et al., 2015). The damage might result due to the disruption of the phospholipid bilayer of cell membrane by the RL owing to its surfactant activity leading to the leakage of electrolytes, protein and DNA (Yan et al., 2015).

*Fusarium verticillioides* has previously been reported to cause seed rot of maize by Yates et al. (2003) wherein a conidial suspension was used to induce seed rot. Therefore, the antifungal activity of RL-SS14 against spores was tested using maize seeds of cv. PAC740 *in vitro*. It was found to be effective in reducing the infection of maize seeds by *F. verticillioides*. The observed antagonistic effect might be due to the inhibitory effect of RL-SS14 against the fungal spores. The findings of this experiment also indicated that RL-SS14 did not have any negative effect on the germination of seeds at the used concentrations. Additionally, *in planta* experiments conducted with RL-SS14 treated seeds also revealed its activity under field conditions as all the seeds treated at a concentration ≥ 50 mg l^-1^ successfully germinated, whereas the untreated seeds failed to germinate in three out of four replicates most likely due to seed rot.

*Fusarium verticillioides* infects maize as a symptomless biotrophic endophyte during most of its association with maize, but under non-ideal culture conditions, the fungus becomes virulent and rapidly colonizes senescing or injured tissue as a saprophyte (Snook et al., 2009). The external symptoms characteristic of *Fusarium* stalk rot include wilting, necrosis at roots, crown or internodes and destruction of pith leading to spongy stalks which can be crushed with little effort. In the present study, RL-SS14 exhibited successful inhibition of stalk rot under controlled conditions during the *in vitro* test using maize stalks.

As *F. verticillioides* causes symptomless infection of stalk and ear of maize, the dry biomass of the plants was evaluated to monitor the comparability of growth to healthy disease free plants. In addition, symptomless stalks were split longitudinally immediately after harvest and cultured in PDA plates to detect the presence of symptomless infection that might account for the reduced biomass of the plants from seeds treated with ≤25 mg l^-1^ RL-SS14. Interestingly, *F. verticillioides* growth was observed from the stalks of plants treated with ≤25 mg l^-1^, while the stalks of plants treated with ≥50 mg l^-1^ did not exhibit any fungal growth. Firstly, this indicates that the endophytic colonization by *F. verticillioides* might have resulted in reduced biomass and absence of fruiting in the plants treated with ≤25 mg l^-1^ and secondly, that RL-SS14 at concentrations ≥ 50 mg l^-1^ successfully inhibited the asymptomatic colonization of the maize stalks by *F. verticillioides*. The treatment with RL-SS14 at concentrations of 50 and 100 mg l^-1^ resulted in improved biomass and fruiting time compared to those of disease free control plants. The seeds treated with 200 mg l^-1^ developed into plants exhibiting comparable biomass and fruiting time with those of healthy plants. In a recent study, Deepika et al. (2015) reported the use of purified RLs produced by *P. aeruginosa* strain KVD-HM52 against *F. oxysporum* in tomato with complete disease inhibition at a concentration of 200 mg l^-1^. The improved performance of the RL-SS14 treated seeds may be attributed to induction of plant resistance as RLs have been reported to elicit defense responses and induce disease resistance (Sanchez et al., 2012). In this regard, RLs have been associated with early events of cell signaling like Ca^2+^ influx, reactive oxygen species (ROS) production and MAP kinase activation along with induction of defense genes associated with pathogenesis related proteins, oxylipins and phytoalexins biosynthesis pathways in grapevine (Varnier et al., 2009). Moreover, biosurfactants have been described to increase the bioavailability of hydrophobic molecules in soil that may serve as nutrients and assist plant growth promotion in the process (Sachdev and Cameotra, 2013). These results highlight the possible use of RL-SS14 as an alternative to chemical surfactants as the use of the latter as adjuvant is a must during the formulation of fungicides (Sachdev and Cameotra, 2013). Jeneil Biosurfactants Co. (Saukville, WI, USA) has successfully commercialized the use of RLs as active compound in the U.S. EPA approved biofungicide Zonix^TM^ (Muller et al., 2012). In a recent study by Johann et al. (2016) involving daphnids and zebrafish embryos, mono-RLs have been described to cause comparable or lower levels of acute toxicity than chemical surfactants and no mutagenic effect confirming their safe use in agricultural and environmental applications.

To conclude, the present study was successful in evaluating the antifungal activity of RL produced by *P. aeruginosa* SS14 against *F. verticilllioides*. The use of 50 mg l^-1^ concentration of RL-SS14 caused complete inhibition of stalk and ear rot disease in maize cv. PAC740 in a single application. No negative effect of RL-SS14 on seed germination and fruiting of the maize cv. was observed in comparison to untreated healthy control plants. On the contrary, the treatment with RL-SS14 at a concentration ≥ 50 mg l^-1^ was observed to improve the fruiting time and biomass of the plants which testify the promising potential of its field application. To our knowledge, this is the first report documenting the use of RL to inhibit *Fusarium* stalk and ear rot and asymptomatic colonization of maize caused by *F. verticillioides* under field conditions.

## Author Contributions

SB designed and carried out the research work, analyzed the data, and wrote the manuscript. DG contributed to the completion of the experiments and the manuscript. HS and SC provided valuable suggestion during the work and manuscript preparation. SD formulated the initial idea and supervised the entire research.

## Conflict of Interest Statement

The authors declare that the research was conducted in the absence of any commercial or financial relationships that could be construed as a potential conflict of interest.

## References

[B1] AbalosA.PinazoA.InfanteM. R.CasalsM.GarciaF.ManresaA. (2001). Physicochemical and antimicrobial properties of new rhamnolipids produced by *Pseudomonas aeruginosa* AT10 from soybean oil refinery wastes. *Langmuir* 17 1367–1371. 10.1021/la0011735

[B2] Abdel-MawgoudA. M.LepineF.DezielE. (2010). Rhamnolipids: diversity of structures, microbial origins and roles. *Appl. Microbiol. Biotechnol.* 86 1323–1336. 10.1007/s00253-010-2498-220336292PMC2854365

[B3] ApSimonJ. W. (2001). Structure, synthesis and biosynthesis of fumonisin B1 and related compounds. *Environ. Health Perspect.* 109 245–249. 10.2307/343501511359692PMC1240672

[B4] BaconC. W.HintonD. M.PorterJ. K.GlennA. E.KuldauG. (2004). Fusaric acid, a *Fusarium verticillioides* metabolite, antagonistic to the endophytic biocontrol bacterium *Bacillus mojavensis*. *Can. J. Bot.* 82 878–885. 10.1139/b04-067

[B5] BorahS. N.DekaS.SarmaH. K. (2016). First report of *Fusarium verticillioides* causing stalk rot of maize in Assam, India. *Plant Dis.* 100 1501 10.1094/PDIS-01-16-0074-PDN

[B6] BorahS. N.GoswamiD.LahkarJ.SarmaH. K.KhanM. R.DekaS. (2015). Rhamnolipid produced by *Pseudomonas aeruginosa* SS14 causes complete suppression of wilt by *Fusarium oxysporum* f. sp. pisi in *Pisum sativum*. *Biocontrol* 60 375–385. 10.1007/s10526-014-9645-0

[B7] CameotraS. S.MakkarR. S.KaurJ.MehtaS. K. (2010). Synthesis of biosurfactants and their advantages to microorganisms and mankind. *Adv. Exp. Med. Biol.* 672 261–280. 10.1007/978-1-4419-5979-9_2020545289

[B8] ConesaA.GötzS.Garcia-GomezJ. M.TerolJ.TalonM.RoblesM. (2005). Blast2GO: a universal tool for annotation, visualization and analysis in functional genomics research. *Bioinformatics* 21 3674–3676. 10.1093/bioinformatics/bti61016081474

[B9] DasP.YangX.-P.MaL. Z. (2014). Analysis of biosurfactants from industrially viable *Pseudomonas* strain isolated from crude oil suggests how rhamnolipids congeners affect emulsification property and antimicrobial activity. *Front. Microbiol.* 5:696 10.3389/fmicb.2014.00696PMC427366025566212

[B10] De JongheK.De DobbelaereI.SarrazynR.HofteM. (2005). Control of *Phytophthora cryptogea* in the hydroponic forcing of witloof chicory with the rhamnolipid-based biosurfactant formulation PRO1. *Plant Pathol.* 54 219–226. 10.1111/j.1365-3059.2005.01140.x

[B11] DeepikaK. V.SridharP. R.BramhachariP. V. (2015). Characterization and antifungal properties of rhamnolipids produced by mangrove sediment bacterium *Pseudomonas aeruginosa* strain KVD-HM52. *Biocatal. Agric. Biotechnol.* 4 608–615. 10.1016/j.bcab.2015.09.009

[B12] DezielE.LepineF.DennieD.BoismenuD.MamerO. A.VillemurR. (1999). Liquid chromatography/mass spectrometry analysis of mixtures of rhamnolipids produced by *Pseudomonas aeruginosa* strain 57RP grown on mannitol or naphthalene. *Biochim. Biophys. Acta* 1440 244–252. 10.1016/S1388-1981(99)00129-810521708

[B13] FeofilovaE. P.SergeevaY. E.MysyakinaI. S.BokarevaD. A. (2015). Lipid composition in cell walls and in mycelial and spore cells of mycelial fungi. *Microbiology* 84 170–176. 10.1134/S002626171502004626263626

[B14] GotzS.Garcia-GomezJ. M.TerolJ.WilliamsT. D.NagarajS. H.NuedaM. J. (2008). High-throughput functional annotation and data mining with the Blast2GO suite. *Nucleic Acids Res.* 36 3420–3435. 10.1093/nar/gkn17618445632PMC2425479

[B15] HabaE.AbalosA.JaureguiO.EspunyM. J.ManresaA. (2003). Use of liquid chromatography-mass spectroscopy for studying the composition and properties of rhamnolipids produced by different strains of *Pseudomonas aeruginosa*. *J. Surfactants Deterg.* 6 155–161. 10.1007/s11743-003-0260-7

[B16] HintonD. M.BaconC. W. (1995). *Enterobacter cloacae* is an endophytic symbiont of corn. *Mycopathologia* 129 117–125. 10.1007/BF011034717659140

[B17] HowardP. C.WarbrittonA.VossK. A.LorentzenR. J.ThurmanJ. D.KovachR. M. (2001). Compensatory regeneration as a mechanism for renal tube carcinogenesis of fumonisin B1 in the F344/N/Nctr BR rat. *Environ. Health Perspect.* 109 309–314. 10.1289/ehp.01109s230911359700PMC1240680

[B18] JohannS.SeilerT. B.TisoT.BluhmK.BlankL. M.HollertH. (2016). Mechanism-specific and whole-organism ecotoxicity of mono-rhamnolipids. *Sci. Total Environ.* 54 155–163. 10.1016/j.scitotenv.2016.01.06626802344

[B19] JurgensonJ. E.ZellerK. A.LeslieJ. F. (2002). Expanded Genetic Map of Gibberella moniliformis (*Fusarium verticillioides*). *Appl. Environ. Microbiol.* 68 1972–1979. 10.1128/AEM.68.4.1972-1979.200211916720PMC123879

[B20] KimB. S.LeeJ. Y.HwangB. K. (2000). In vivo control and in vitro antifungal activity of rhamnolipid B, a glycolipid antibiotic, against *Phytophthora capsici* and *Colletotrichum orbiculare*. *Pest Manage. Sci.* 56 1029–1035. 10.1002/1526-4998(200012)56:12<1029::AID-PS238>3.0.CO;2-Q

[B21] LahkarJ.BorahS. N.DekaS.AhmedG. (2015). Biosurfactant of *Pseudomonas aeruginosa* JS29 against *Alternaria solani*: the causal organism of early blight of tomato. *BioControl* 60 401–411. 10.1007/s10526-015-9650-y

[B22] MagalhaesL.NitschkeM. (2013). Antimicrobial activity of rhamnolipids against Listeria monocytogenes and their synergistic interaction with nisin. *Food Control.* 29 138–142. 10.1016/j.foodcont.2012.06.009

[B23] MarasasW. F. O. (2001). Discovery and occurrence of fumonisins: a historical perspective. *Environ. Health Perspect.* 109 239–243. 10.2307/343501411359691PMC1240671

[B24] MarasasW. F. O.RileyR. T.HendricksK. A.StevensV. L.SadlerT. W.van WaesJ. G. (2004). Fumonisins disrupt sphingolipid metabolism, folate transport, and neural tube development in embryo culture and in vivo: a potential risk factor for human neural tube defects among populations consuming fumonisin contaminated maize. *J. Nutr.* 134 711–716.1505181510.1093/jn/134.4.711

[B25] MullerM. M.KuglerJ. H.HenkelM.GerlitzkiM.HormannB.PohnleinM. (2012). Rhamnolipids-next generation surfactants? *J. Biotechnol.* 162 366–380. 10.1016/j.jbiotec.2012.05.02222728388

[B26] MunkvoldG. P.DesjardinsA. E. (1997). Fumonisins in maize. can we reduce their occurrence? *Plant Dis.* 81 556–564. 10.1094/PDIS.1997.81.6.55630861834

[B27] MunkvoldG. P.HellmichR. L.RiceL. G. (1998). Comparison of fumonisin concentrations in kernels of transgenic Bt-maize hybrids and nontransgenic hybrids. *Plant Dis.* 83 130–138. 10.1094/PDIS.1999.83.2.13030849794

[B28] MunkvoldG. P.HellmichR. L.ShowersW. B. (1997). Reduced *Fusarium* ear rot and symptomless infection in kernels of maize genetically engineered for European corn borer resistance. *Phytopathology* 87 1071–1077. 10.1094/PHYTO.1997.87.10.107118945043

[B29] NitschkeM.CostaS. G. V. A. O. (2007). Biosurfactants in food industry. *Trends Food Sci. Tech.* 18 252–259. 10.1016/j.tifs.2007.01.002

[B30] PalmeroD.Gil-SernaJ.GalvezL.CurtM. D.De CaraM.TeloJ. (2012). First report of *Fusarium verticillioides* causing stalk and root rot of *Sorghum* in Spain. *Plant Dis.* 96 584 10.1094/PDIS-11-11-0958-PDN30727442

[B31] PerneelM.D’hondtL.De MaeyerK.AdioboA.RabaeyK.HofteM. (2008). Phenazines and biosurfactants interact in the biological control of soil-borne diseases caused by *Pythium* spp. *Environ. Microbiol.* 10 778–788. 10.1111/j.1462-2920.2007.01501.x18237310

[B32] PiljacT.PiljacG. (2007). Use of rhamnolipids as Cosmetics. EP 1056462B1.

[B33] PornsunthorntaweeP.WongpanitP.ChavadejS.AbeM.RujiravanitR. (2008). Structural and physicochemical characterization of crude biosurfactant produced by *Pseudomonas aeruginosa* SP4 isolated from petroleum-contaminated soil. *Bioresour. Technol.* 99 1589–1595. 10.1016/j.biortech.2007.04.02017540558

[B34] RahmanK. S. M.RahmanT. J.KourkoutasY.PetsasI.MarchantR.BanatI. M. (2003). Enhanced bioremediation of n-alkane in petroleum sludge using bacterial consortium amended with rhamnolipid and micronutrients. *Bioresour. Technol.* 90 159–168. 10.1016/S0960-8524(03)00114-712895559

[B35] RandhawaK. K. S.RahmanK. S. M. (2014). Rhamnolipid biosurfactants – past, present, and future scenario of global market. *Front. Microbiol.* 5:454 10.3389/fmicb.2014.00454PMC415138225228898

[B36] RheederJ. P.MarasasW. F. O.ThielP. G.SydenhamE. W.ShephardG. S.van SchalkwykD. J. (1992). *Fusarium* moniliforme and fumonisins in corn in relation to human esophageal cancer in Transkei. *Phytopathology* 82 353–357. 10.1094/Phyto-82-353

[B37] SachdevD. P.CameotraS. S. (2013). Biosurfactants in agriculture. *Appl. Microbiol. Biotechnol.* 97 1005–1016. 10.1007/s00253-012-4641-823280539PMC3555348

[B38] SaitouN.NeiM. (1987). The neighbor-joining method: a new method for reconstructing phylogenetic trees. *Mol. Biol. Evol.* 4 406–425.344701510.1093/oxfordjournals.molbev.a040454

[B39] SanchezL.CourteauxB.HubertJ.KauffmannS.RenaultJ. H.ClementC. (2012). Rhamnolipids elicit defense responses and induce disease resistance against biotrophic, hemibiotrophic, and necrotrophic pathogens that require different signaling pathways in *Arabidopsis* and highlight a central role for salicylic acid. *Plant Physiol.* 160 1630–1641. 10.1104/pp.112.20191322968829PMC3490604

[B40] ShaR.JiangL.MengQ.ZhangG.SongZ. (2012). Producing cell-free culture broth of rhamnolipids as a cost-effective fungicide against plant pathogens. *J. Basic Microbiol.* 52 458–466. 10.1002/jobm.20110029522052667

[B41] SharmaP. (2011). Alarming occurrence of *Fusarium* wilt disease in pea (*Pisum sativum* L.) cultivations of Jabalpur district in Central India revealed by an array of pathogenicity tests. *Agric. Biol. J. N. Am.* 2 981–994. 10.5251/abjna.2011.2.6.981.994

[B42] SnookM. E.MitchellT.HintonD. M.BaconC. W. (2009). Isolation and characterization of Leu7-surfactin from the endophytic bacterium *Bacillus mojavensis* RRC 101, a biocontrol agent for *Fusarium verticillioides*. *J. Agric. Food Chem.* 57 4287–4292. 10.1021/jf900164h19371139

[B43] TamuraK.StecherG.PetersonD.FilipskiA.KumarS. (2013). MEGA6: molecular evolutionary genetics analysis version 6.0. *Molecul. Biol. Evol.* 30 2725–2729. 10.1093/molbev/mst197PMC384031224132122

[B44] VarnierA. L.SanchezL.VatsaP.BoudesocqueL.Garcia-BruggerA.RabenoelinaF. (2009). Bacterial rhamnolipids are novel MAMPs conferring resistance to *Botrytis cinerea* in grapevine. *Plant Cell Environ.* 32 178–193. 10.1111/j.1365-3040.2008.01911.x19021887

[B45] WeiY. H.ChoubC. L.ChangJ. S. (2005). Rhamnolipid production by indigenous *Pseudomonas aeruginosa* J4 originating from petrochemical wastewater. *Biochem. Eng. J.* 27 146–154. 10.1016/j.bej.2005.08.028

[B46] WuJ. Y.YehK. L.LuW. B.LinC. L.ChangJ. S. (2008). Rhamnolipid production with indigenous *Pseudomonas aeruginosa* EM1 isolated from oil-contaminated site. *Bioresour. Technol.* 99 1157–1164. 10.1016/j.biortech.2007.02.02617434729

[B47] YanF.XuS.GuoJ.ChenQ.MengQ.ZhengX. (2015). Biocontrol of post-harvest *Alternaria alternata* decay of cherry tomatoes with rhamnolipids and possible mechanisms of action. *J. Sci. Food. Agric.* 95 1469–1474. 10.1002/jsfa.684525065672

[B48] YatesI. E.ArnoldJ. W.HintonD. M.BasingerW.WalcottR. R. (2003). *Fusarium verticillioides* induction of maize seed rot and its control. *Can. J. Bot.* 81 422–428. 10.1139/B03-034

